RETRACTED

# Oral Haemangioma

**DOI:** 10.1155/2012/347939

**Published:** 2012-02-06

**Authors:** Jaspreet Singh Gill, Sharanjeet Gill, Amit Bhardwaj, Harpreet Singh Grover

**Affiliations:** ^1^Department of Periodontics and Oral Implantology, SGT Dental College, Hospital and Research Institute, Gurgaon, Budhera, Haryana 122505, India; ^2^Department of Oral Pathology, Manav Rachna Dental College, Haryana, Faridabad 121004, India

## Abstract

Vascular anomalies comprise a widely heterogeneous group of tumours and malformations. Haemangioma is the most common benign tumour of vascular origin of the head and neck region. The possible sites of occurrence in oral cavity are lips, tongue, buccal mucosa, and palate. Despite its benign origin and behaviour, it is always of clinical importance to the dental profession and requires appropriate management. This case study reports a rare case of capillary haemangioma on the palatal gingiva in a 14-year-old female.

## 1. Introduction

Haemangioma are the most common benign vasoformative tumours of infancy and childhood [1, 2]. They usually are manifested within the first month of life, exhibit a rapid proliferative phase, and slowly involute to near complete resolution. There are many ways to classify haemangiomas. According to Enzinger and Weiss, haemangiomas are broadly classified into capillary, cavernous, and miscellaneous forms like verrucous, venous, arteriovenous haemangiomas, and so forth [3]. Capillary haemangiomas further include juvenile, pyogenic granuloma, and epitheliod haemangioma [3]. The term haemangioma has been commonly misused to describe a large number of vasoformative tumours [4]. However, the International Society for the Study of Vascular Anomalies (ISSVA) has recently provided guidelines to differentiate these two conditions, according to the novel classification first published by Mulliken et al. in 1982 [5]. Vasoformative tumours are broadly classified into two groups: haemangioma and vascular malformation [5]. Haemangioma is histologically further classified into capillary and cavernous forms [6, 7]. Capillary haemangioma is composed of many small capillaries lines by a single layer of endothelial cells supported in a connective tissue stroma of varying density, while cavernous haemangioma is formed by large, thin walled vessels, or sinusoids lined by epithelial cells separated by thin layer of connective tissue septa [8].

The majority of haemangioma involve the head and neck. However, they are rare in the oral cavity but may occur on tongue, lips, buccal mucosa, gingiva, palatal mucosa, salivary glands, alveolar ridge, and jaw bones [3, 4, 6, 9–12]. Clinically, haemangioma appears as soft mass, smooth or lobulated, and sessile or pedunculated and may vary in size from a few mms to several cms [8]. They are usually deep red and may blanch on the application of pressure and if large in size, might interfere with mastication [9]. In the present case study, we report a rare and an unusual case of capillary haemangioma of the palatal mucosa.

RETRACTED

## 2. Case Report

A female patient aged 14 years, reported with a chief complaint of a swelling and growth on the inner side of her upper front teeth since 4-5 months. She also complains of localized bleeding in that area on brushing, and there was slight pain and discomfort on eating.

Dental history revealed that she had a history of gingival enlargement, one year back, which she had got excised. However, the growth recurred within two months after surgical excision. It was initially small in size, gradually increased and stabilized after 3-4 weeks till the present size. On general physical examination, it was found that the patient was normally built for her age with no defect in gait or stature, and there was no relevant medical history. Family history was also noncontributory.

A comprehensive intraoral examination revealed a localized gingival mass between maxillary right central incisor and lateral incisor (11, 12) on the palatal aspect (Figure 1). It was firm, pedunculated with a distinct stalk arising from the interdental papillary region. The mass was bright red, erythematous and bilobulated with well-defined margins. The two distinct lobes measured about 5 cm × 4 cm and 3 cm × 2.5 cm in diameter. They were firm and rubbery in texture. No surface ulceration or secondary infection was noted. Periodontal examination revealed no clinical attachment loss. Panoramic examination confirmed no alveolar bone loss, and a provisional diagnosis of pyogenic granuloma was made on the basis of history and clinical features.

The other pathologic entities that were included in the differential diagnosis were malignancies, trauma, and or infection (bacterial, viral, and fungal), enlargement due to drugs. Complete blood examination, urine analysis, and an intraoral periapical radiograph with respect to 11, 12 were done. The laboratory investigations of blood and urine were within normal limits that ruled out any leukemic enlargement and diabetes mellitus. HIV, HBs, VDRL, and Mantoux test were negative, ruling out any possibility of infectious involvement. Radiographically, there was no evidence of crestal bone loss, and lamina dura was intact around the roots of both maxillary right central and lateral incisor. Scaling was carried out under universal precautions, and later surgical excision of the lesion was done under local anaesthesia as a part of excisional biopsy. A thread was tied around the stalk of the pedunculated lesion and was stretched tightly so as to reduce blood circulation to the lesion. The growth was then surgically excised along with the stalk, and thorough curettage of the area was performed. The excised lesion was stored in 10% formalin and sent for histopathological examination. Periodontal dressing was applied on the operated area, and the patient was given postoperative instructions. Histopathological examination revealed stratified squamous epithelium which showed atrophy, and in some areas hyperkeratosis was seen. Beneath this, many small and large capillaries filled with blood were present. These vessels were lined by a single layer of endothelial cells and were supported by a connective tissue stroma of varying density with no inflammatory component (Figure 2). On the basis of clinical examination and histopathology, a diagnosis of capillary haemangioma was made. The patient was recalled after a week with normal healing and various plaque control measures were reinforced (Figure 3). The patient was also reviewed 1, 3, and 6 months after the biopsy, and there was no recurrence of the lesion.

RETRACTED

## 3. Discussion

The confusing and misleading terminology has led to inappropriate grouping and classification of vasoformative tumours [4]. The differentiation between haemangioma and vascular malformations is made on the basis of clinical appearance, histopathology, and biological behaviour [4].

Pathogenesis and origin of haemangioma remain incompletely understood. However, various theories have been proposed to elucidate the mechanism and pathogenesis of haemangioma. Aberrant and focal proliferation of endothelial cells results in haemangioma, although the cause behind this remains unclear [13]. The placental theory of haemangioma origin has been described by North et al. [14], who studied various histology and molecular markers such as GLUTI, Lewis Y Antigen, Merosin, CCR6, CD15, IDO, FC, and gamma Receptor II. Positive staining for GLUTI is considered highly specific and diagnostic for haemangioma, and it is useful for making differential diagnosis between haemangioma and other vascular lesions clinically related to it [13]. More recently, somatic mutational events in gene involved in angiogenesis are related to haemangioma growth [4]. Growth factors specifically involved in angiogenesis such as VEGF, b-TGF, and IGF are often increased during the proliferation phases of haemangioma growth [15, 16]. Moreover, it has been noted that during the involution phase of haemangioma, there is a decrease in angiogenic molecules (VEGF, PCNA, Type IV collagenase, Lewis V antigen, CD 31), while there is increase in concentration of marker for apoptosis (T4, TUNNEL, INF, Mast cells, and TGF) [4, 17, 18]. Thus, role of molecular signalling is now clear in haemangioma development.

RETRACTED

A variety of other lesions can resemble haemangioma in the oral cavity. The differential diagnosis includes pyogenic granuloma, chronic inflammatory gingival hyperplasia, epulis granulomatosa, telangiectasia, angiosarcoma, squamous cell carcinoma, and other vascular appearing lesions of face or oral cavity such as Sturge Weber Syndrome [9].

In the present case, clinical features resemble that of pyogenic granuloma. However, the lesion did not show microscopic appearance of a pyogenic granuloma. It contained blood-filled capillaries lined by layer of endothelial cells in a connective tissue stroma without any evidence of inflammation.

Angiosarcoma is a rare malignant tumour of vascular endothelium, and it resembles haemangioma. However, it can be differentiated from it on the basis of histopathologic findings as it is characterized by infiltrative proliferation of endothelium-lined blood vessels that form an anastomosing network. The endothelial cells appear hyperchromatic and atypical and often tend to pile up within vascular lamina [8].

Management of haemangioma depends on a variety of factors, and most true haemangioma requires no intervention. However, 10–20% requires treatment because of the size, exact location, stages of growth or regeneration, functional compromise, and behaviour. The range of treatment includes surgery, flash lamp pulsed laser, intralesional injection of fibrosing agent, interferon alpha-2b, and electrocoagulation while cryosurgery, compression and radiation were used in the past [11–13, 19–22]. Each treatment modality has its own risk and benefits. In the present case, surgery was carried out on the basis of size and location. Moreover, the difficulty in swallowing was another factor that was taken in consideration, and surgical approach was preferred as to remove excess residual fibrofatty and redundant tissue after involution.

## 4. Conclusion

Haemangioma is of benign origin and behaviour, but haemangioma in the oral cavity is of clinical importance. It often mimics other lesion clinically and requires appropriate clinical diagnosis and proper management.

## Figures and Tables

**Figure 1:** Preoperative intraoral view.

**Figure 2:** H and E stain section at 10x magnification showing numerous blood-filled capillaries in connective tissue stroma.

**Figure 3:** Postoperative view after one week.
